The article "Application of CT Multimodal Images in Rehabilitation Monitoring of Long-Distance Running" was retracted in 2023. Reasons: signs of a paper mill; compromised peer review; unreliable results or conclusions.

# Application of CT Multimodal Images in Rehabilitation Monitoring of Long-Distance Running

**DOI:** 10.1155/2022/6425448

**Published:** 2022-10-04

**Authors:** Xufeng Du, Yaye He

**Affiliations:** ^1^Physical Education Department of Shanxi Medical University, Taiyuan Shanxi 030001, China; ^2^Science and Education Department Taiyuan Central Hospital, Taiyuan Shanxi 030001, China

## Abstract

In order to monitor the rehabilitation of athletes injured in long-distance running, the author proposes a method for rehabilitation monitoring of long-distance running based on CT multimodal images. This method combines the latest multimodal image technology, integrates multimodal technology into CT images to improve the accuracy, performs image segmentation on CT multimodal images through medical segmentation methods, and analyzes the segmented images; finally, it can achieve the effect of rehabilitation treatment for athletes in long-distance running. Experimental results show that the total time taken by the authors' method is 10.9 hours, with an average time of 8 seconds, which is much shorter than the other two control methods. In conclusion, the authors' method allows for better rehabilitation monitoring of long-distance running sports injuries.

## 1. Introduction

Middle-distance running is short for middle-distance running and long-distance running [1]. In middle- and long-distance running, athletes may cause sports injuries due to the consumption of energy substances in the body and the accumulation of metabolites, the decline of exercise ability, technical deformation, and weak awareness of self-protection. Therefore, it is of great significance to study the causes and preventive measures of injuries in middle- and long-distance running; at the same time, the rehabilitation monitoring of the injured part is also very important [2, 3].

In recent years, with the continuous development of the mobile Internet and the continuous popularization of multimedia and smart portable devices, more and more information such as images, voices, and texts are stored on the network and smart devices in the form of data. Images and videos have become another main information carrier after text; now, billions of images are uploaded every day; in the future, there will be a lot of search work related to images and videos; therefore, machines automatically understand image semantics and establish a relationship between images and texts; the relationship between them has become a research topic of practical significance. In recent years, various university laboratories, research institutions, and company laboratories have been carrying out this research in depth. Based on deep learning, researchers have conducted in-depth research on applications in computer vision and natural language processing and achieved excellent results. Multimodal image understanding (image description), as a high-level image semantic understanding task, also involves multimodal problems related to computer vision and natural language processing and is an important exploration for the application of deep learning to multiple modal fields [4].

Medical image segmentation is the basis of medical image processing and analysis, the solution of this problem not only directly affects the successful application of computer graphics and image technology in medicine but also has important theoretical and practical significance [5–7]. Medical image segmentation is a process of extracting regions of interest, and the segmentation results can provide reference for subsequent disease diagnosis, treatment plan planning, and treatment effect evaluation. Because of its high resolution, CT can more clearly highlight the characteristics of anatomical structure and diseased tissue, which makes it widely used in the diagnosis of diseases in many systems. Therefore, it is very important to study the application of image segmentation methods in CT images, as shown in Figure 1.

## 2. Literature Review

With the increase of competition intensity and the improvement of athletes' competitive level, the training intensity of middle-distance runners is also increasing. However, due to the relatively weak awareness of self-protection of athletes, sports injuries occur from time to time. There are five common injuries:

1. Overuse injury
2. Joint sprain
3. Strain
4. Abdominal pain during exercise
5. Muscle spasm

For these five kinds of injuries, relevant parties have made rehabilitation methods for these five methods and achieved ideal therapeutic effects. But it does not apply to all types of damage.

The multimodal image understanding task can be applied in many aspects and has strong practicality [8]. For example, it can be used for search functions, including image-text search and text-image search, so that the traditional tag-based search is converted into a tag and content-based search, and the search results are more accurate; at the same time, the search time is saved, and it has high practical significance. Multimodal image understanding can also be used for assistive functions, specifically assisting those systems without visual systems or visually impaired, such as intelligent robots assisting the blind; the robot can observe the external environment according to the visual system and convert it into text information is described, then use speech synthesis technology to achieve text-to-speech conversion, so as to better help visually impaired people, and can also be used in early childhood education; multimodal image understanding technology can teach children to see pictures and speak, and at the same time, in medical imaging, multimodal image understanding technology can automatically generate diagnostic results and assist doctors in seeing patients. Therefore, the multimodal image understanding task has a wide range of application scenarios in real life and has extremely high academic value and research significance that cannot be ignored in scientific research [9].

The current mainstream solutions for multimodal image understanding tasks are based on encoder-decoder frameworks. For example, Teng and Wu use an encoder to encode an input image and a decoder to generate captions for the image [10]. Among them, the common encoder is a deep convolutional neural network, and the decoder often uses an autoregressive decoder such as a recurrent neural network, such as LSTM; the autoregressive decoder sequentially generates each word in a serialized manner, resulting in a complete descriptive sentence. Since the autoregressive decoder is based on the previously generated word sequence and image content to generate the words of the current time step, this is a serialization process, which cannot be parallelized, so there is a problem of slow generation speed. Moreover, in the process of generating words by reasoning, if the previous words are inappropriate or there is a deviation error, it is easy to affect the words generated later, resulting in cumulative errors. At the same time, the autoregressive decoder treats the sentence as a serialized structure instead of a hierarchical structure, this process cannot model the inherent hierarchical structure of natural language, and this makes the autoregressive decoder extremely favor N-gram phrases with high frequency in the training data and is more inclined to predict common phrases [11]. Therefore, autoregressive decoders run the risk of incorrect semantics and lack of sentence diversity. In the neural machine translation model (NMT), the nonautoregressive decoder is proposed to solve the problem that the generation speed of the autoregressive decoder is too slow, but this nonautoregressive decoder indirectly models the real target modal distribution, rather than modeling its distribution directly. Direct modeling follows the conditional generation method of language, that is, it predicts the word at the current moment based on the condition of the sentence above, and the autoregressive decoder adopts the direct modeling method. Indirect modeling follows the condition-independent generation method of language, that is, each word in the entire sentence is independently generated without being conditioned on the context. Therefore, indirect modeling does not follow the conditional distribution of the language, which inevitably introduces another problem, called the “multimodal problem.”

CT has created a precedent for digital imaging, but it is different from ordinary X-ray imaging. CT displays sectional anatomical images, and its density resolution capability is much higher than that of X-ray images, so that X-ray imaging cannot develop anatomical structures and their lesions. Organization is visualized; thus, the inspection scope of the human body is significantly expanded, and the detection rate of lesions and the accuracy of diagnosis are improved. As the first digital imaging device developed, CT has greatly promoted the development of medical imaging. At present, CT has been widely used in the diagnosis of the following systems and organ diseases in clinic: central nervous system, head and neck, lungs, heart and great vessels, abdomen and pelvis, and musculoskeletal system.

Based on the above research, the author proposes a rehabilitation monitoring method for long-distance running sports injuries based on CT multimodal images. Combining CT medical segmentation technology and multimodal image technology, we form a CT multimodal image technology and use CT image cutting technology and multimodal image technology to medically cut and analyze CT multimodal images; this not only achieves the use of CT images for the rehabilitation of long-distance running injuries but also speeds up the monitoring speed and improves the rehabilitation effect.

## 3. Research Methods

### 3.1. Multimodal Image Understanding Model

The algorithm of multimodal image understanding model mainly includes algorithm based on template matching, search, and multimodal image understanding based on neural network. The method based on template matching first recognizes visual elements such as objects existing in it, the relationship between objects, scene locations, etc. through scene recognition and target monitoring, then fill in the sentence template designed by hand; the disadvantage is that the sentence pattern is fixed, the generated sentence is too simple and lacks flexibility, and at the same time, this method requires identifying the relationship between objects, scene content, and objects in advance; the workload is large in the early stage, which will overrely on the performance of the experiment, and is prone to error accumulation; this is a way of inducing biases directly using the dataset. The search-based algorithm is used to search for similar images in the training dataset, and the description sentence of the most similar image is used as the description sentence of the image; compared with the template matching method, the sentences generated by this method are more fluent. The disadvantage is that similar pictures will have different content, so it is difficult to generate accurate sentences describing the images. The sentences generated by these methods are relatively simple and have a high error rate. For this reason, many researchers are constantly exploring new solutions, including multimodal image understanding models based on neural networks. The following will mainly introduce the multimodal image understanding model based on neural network.

The current popular algorithms for multimodal image understanding models are mainly based on deep neural network algorithms, inspired by the successful application of neural network training in machine translation; such algorithms usually use an encoder-decoder framework. The specific process is as follows: Use an encoder (such as a convolutional neural network CNN) to extract the features of the image, and then use a decoder (such as a recurrent neural network LSTM) to decode the image features into smooth sentences. At prediction time, each step of the LSTM generates a word until a period is generated. Here, the word predicted at the previous moment and the internal state are input into LSTM, and then LSTM predicts the distribution of words and takes the word with the highest probability as the word at this moment. During training, a supervised method is generally used, so pairs of images and text are required. The input of each moment of LSTM is the word of the correct text at the previous moment, and then the probability of the word of the correct text at this moment is optimized. This is a calculation method of maximum likelihood estimation, which increases the probability of text in the dataset. This model breaks through the confinement of traditional multimodal image understanding and achieves high scores in various evaluation indicators, laying a theoretical guide for today's multimodal image understanding models.

### 3.2. Theories Related to CT Images

#### 3.2.1. CT Images and CT Values

A CT image consists of two parts: the intensity and size of the pixel, where the intensity of the pixel reflects the absorption of X-rays by the organ or tissue, and the size of the pixel reflects the fineness of the image, that is, the spatial resolution of the image [12]. In the process of CT imaging, the measurement accuracy of the X-ray absorption coefficient of organs or tissues can reach 0.5%. Therefore, compared with X-ray images, CT images have higher density resolution. In reality, for the convenience of expression, the CT value is usually used instead of the absorption coefficient to express the degree of X-ray absorption by an organ or tissue.

Figure 2 shows the CT values corresponding to various tissues of the human body. A careful study of the figure shows that the CT value corresponding to the bone is the highest, the CT value corresponding to the air is the lowest, and the CT value of the other tissues of the human body is in between.

#### 3.2.2. CT Slice

CT images are three-dimensional images of the human body, and CT images are often observed and analyzed from different directions in practical applications [13]. In human anatomy, the section that cuts the human body into two parts longitudinally along the left and right directions is called the coronal plane. The plane passing through the vertical axis and longitudinal axis of the human body and all parallel planes are called sagittal planes. The surface exposed after cutting the human body perpendicular to the axis of the human body is called the transverse plane.

#### 3.2.3. Research Characteristics of CT Image Segmentation Methods

Compared with general images, CT images have the characteristics of anatomical tissue structure and shape complexity, inherent ambiguity of the image, inhomogeneity of grayscale within the tissue, and massive data. Therefore, the research on CT image segmentation methods correspondingly presents the following characteristics: (1) Due to the potential complexity and diversity of CT images and the difficulty of the segmentation problem itself, so far, there is no segmentation method that can be applied to various tasks, and it is usually the right segmentation for a specific task algorithm. Furthermore, due to the limitations of various segmentation methods, people are trying to explore new methods for CT image segmentation and pay more attention to the combination of multiple segmentation methods. (2) Although the obtained CT images exist in the form of two-dimensional slices, with the improvement of computer performance, the research on three-dimensional segmentation methods has received more and more attention; the reason is that the integrity of human organs ensures the continuity of CT images of adjacent slices, so the 3D segmentation method can use more information between slices to guide the segmentation process, making the segmentation results more accurate. (3) Medical images can be divided into anatomical images and functional images according to their functions, the former mainly describes human anatomical information, while the latter mainly describes human function and metabolic information. CT images belong to anatomical images. In the process of CT image segmentation, it has gradually become a new trend to fuse other functional images, such as positron emission tomography images, in order to guide CT image segmentation [14]. (4) Image segmentation algorithms can be divided into three categories according to their degree of automation: automatic, interactive, and manual segmentation [15–17]. Due to the increasing precision of modern instruments, the volume of CT data is increasing, making manual segmentation almost impossible, and the results of manual segmentation have a lot to do with the experience of the operator; at the same time, the results are not repeatable, which greatly limits its application. Therefore, automatic segmentation is the goal of the segmentation algorithm design process. However, the complexity of the CT image itself makes the current automatic segmentation algorithms have achieved some successes, but they are far from meeting the requirements for the accuracy of the results in the process of clinical practical application. Therefore, user-initiated and user-guided interactive CT image segmentation methods have received more and more attention. The human-machine interactive segmentation method can not only give play to the subjective initiative of people; therefore, the accuracy of the segmentation algorithm is ensured, and the performance of the computer can be fully utilized, thereby ensuring the practicability of the segmentation algorithm

### 3.3. Multimodal Image Segmentation of Hip CT Based on Adaptive Classification and Normal Direction Correction

#### 3.3.1. Image Initial Segmentation

After preprocessing the hip CT multimodal image, the initial segmentation of the image consists of two steps, the first step is to binarize the image using the global optimal threshold method [18]. Due to the higher density of bone relative to its surrounding soft tissue, bone has a higher intensity than the surrounding soft tissue in CT multimodal images. The threshold method is often used as the preferred method for rough bone segmentation due to its simple operation and high algorithm execution efficiency [19]. In the binarized image, the approximate area of the bone has been segmented, but due to the nonuniformity of bone density and the existence of lesions in the bone, the threshold method often causes holes in the bone in the binarized image, and bone boundaries produce discontinuities. In view of the above problems, in the second step, the 3D mathematical morphology method is used to fill the holes and connect the boundaries of the binarized images.

#### 3.3.2. Histogram-Based Thresholding

The segmentation of the hip joint is achieved using a multistep method, and the basic steps are to first perform an initial segmentation of the CT multimodal images; then we use this segmentation result to initialize the iterative adaptive segmentation algorithm to achieve complete separation of bone and nonbone tissue and finally use the normal direction correction algorithm to achieve accurate positioning of the bone boundary.

There are many methods for initial segmentation of bone, such as threshold method, serpentine method, region growth method, watershed segmentation method, etc. Compared with other segmentation methods, threshold segmentation method is one of the most commonly used bone CT image segmentation methods, the reason is that in CT multimodal images, the bone tissue generally has a higher density than the surrounding soft tissue, and the threshold method can be used to achieve a simple and fast segmentation of the bone, then realizing the fast initialization of the iterative adaptive classification process; thereby, the execution efficiency of the whole algorithm is improved; due to the large amount of computation, the efficiency of other methods is much lower than that of threshold segmentation [20].

The advantage of threshold segmentation is that it is simple and fast. When the gray value of objects belonging to different types or their eigenvalues are very different, it can effectively segment the objects. The thresholding segmentation method mainly includes two steps:

1. Determine the required segmentation threshold
2. Compare the segmentation threshold with the voxel gray value to divide the voxels

In the above steps, determining the threshold is the key to segmentation. When using the threshold method to segment a grayscale image, there are generally certain assumptions about the image. In other words, it is based on a certain image model, for example, it is assumed that the gray distribution of different categories in the image conforms to the Gaussian distribution. Specifically applied to the CT multimodal image of the hip joint, considering that the bone has a significantly higher intensity than other soft tissues, and the internal intensity of the soft tissue does not change much, the gray histogram of the hip joint can basically be regarded as composed of a mixture of two unimodal histograms corresponding to bone tissue and soft tissue.

For the grayscale histogram composed of the mixture of two unimodal histograms, the author determines the initial segmentation threshold according to the Otsu algorithm. The basic idea of Otsu algorithm is to find a threshold; this threshold maximizes the between-class variance and, at the same time, minimizes the within-bird variance. According to the theory of discriminant analysis, such a threshold is the optimal segmentation threshold.

The specific steps for determining the optimal threshold are as follows: Firstly, calculate the grayscale histogram of the region of interest (ROI) of the hip joint. Since the CT value of soft tissue is smaller than that of bone tissue and the number of soft tissue voxels in the ROI accounts for a larger proportion, therefore, it can be judged from the histogram that high peaks correspond to soft tissue types, and low peaks correspond to bone tissue types. In this chapter, it is assumed that both soft tissue and bone tissue obey the Gaussian distribution. During the calculation of the optimal threshold, two Gaussian curves are used to fit the histogram curve; it can be known that the gray value corresponding to the intersection of the two Gaussian curves is the optimal segmentation threshold, as shown in Figure 3.

#### 3.3.3. Binary Image Morphological Operations

In the binary image obtained by the above thresholding method, there are often holes in the bone tissue, discontinuity at the edge of the bone, and wrong connection between the bones. These phenomena are due to the nonuniformity of bone tissue density, the weak edge nature of bone, and the partial volume effect during CT multimodal imaging. In order to roughly obtain the bone tissue area for subsequent accurate edge segmentation, the author uses mathematical morphology to fill the “holes” in the obtained binary image. In general, the choice of structural elements (size and shape) affects the results of morphological operations. Commonly used structuring element shapes are sphere, cube, and rhombus. In order to minimize bone-to-bone misconnections due to morphological methods, the authors took 3 × 3 × 3 diamond-shaped structural elements.

#### 3.3.4. Iterative Reclassification Algorithm Computation

*(1) Calculate the Bone Boundaries from the Current Segmentation*. For a given voxel, if its directly connected neighbor voxels can be divided into two different classes, the voxel is located at the edge of the bone area *B* or the nonbone area *B*. In order to calculate the voxels of the bone edge, a six-voxel neighborhood structure is first defined, and the voxel set of the spine edge in this chapter is *E*. Specifically, for each voxel *x* in *B*, if any one of its six neighboring voxels belongs to $\bar{B}$, then the voxel belongs to the set *E*_*B*_. For the convenience of the following description, the authors here specifically label voxels *x* belonging to set *E*_*B*_ as *x*^∗^.

#### 3.3.5. Reclassification of Bone Boundary Regions Based on Bayesian Decision Criteria

For each bounding voxel *x*, first define a window *W*(*x*^∗^) centered on the position of *x*. All voxels in *W*(*x*^∗^) are assumed to be derived from two Gaussian distributions (bone region *B* and nonbone Region $\bar{B}$) with mean and standard deviation (*μ*_1_, *σ*_1_) and (*μ*_2_, *σ*_2_), respectively. For convenience, note *φ*_1_=(*μ*_1_, *σ*_1_), *φ*_2_=(*μ*_2_, *σ*_2_). The estimation method of parameters *φ*_1_, *φ*_2_ will be discussed in detail later Figure 4.

According to Bayes' theorem, for a given voxel *x*, the proportion of bone components in the voxel can be calculated by the following formula:

(1) $$\begin{array}{c} p\left(a^{x}\left|y_{x}\right.\right)=\frac{p\left(y_{x}\left|a^{x}\right.\right)p\left(a^{x}\right)}{p\left(y_{x}\right)}. \end{array}$$

#### 3.3.6. Update the Current Segmentation Result

After each voxel in *E*_*B*_ has been traversed, the new bone area *B* and nonbone area $\bar{B}$ are obtained again by using the three-dimensional mathematical morphology method. After the new bone and nonbone areas are obtained, the boundary voxel set *E*_*B*_ will be recalculated. If the voxels in *E*_*B*_ do not change during the two iterations before and after, the iteration process will be stopped. Otherwise, turn to the first step to recalculate the bone boundary voxels and perform the entire iterative process until convergence.

## 4. Results and Discussion

The authors conducted a retrospective analysis of the experimental results. In this experiment, 55 sets of CT multimodal data images were collected, including a total of 110 hip joints. The experimental data comes from a GE Pro Speed CT machine, the slice plane resolution is 512 × 512, the in-plane pixel pitch is 0.68 mm, the distance between slices is 1.5 mm, and the number of slices is 85 to 95. The experimental environment is MATLAB6.5, 2.33 GHz processor, 2 GB memory. Among the 110 hip joints, data ranging from normal to severe lesions were included. Manual segmentation results of all data were given by radiologists.

In order to verify the applicability of the proposed method, the authors based on anatomical and imaging features (e.g., the proximity of the femoral head to the acetabulum, the degree of deformity of the femoral head, and the degree of inhomogeneity of bone density); the obtained 110 hip joints were divided into four groups, and the numbers of the four groups were 16, 31, 51, and 12, respectively. Further research can be found that this method belongs to the model-based segmentation method; in the segmentation process, the shape information of the object to be segmented is added as a priori constraint knowledge; therefore, the segmentation method is more robust for hip joints with severe lesions.  Table 1 shows the comparison results of this method and the other two methods in terms of segmentation time.

It can be seen that the author's method takes a total of 10.9 hours, and the average time is 8 seconds, which is much shorter than the other two methods, indicating that the author's method has great advantages in the field of image segmentation. Therefore, the injuries caused by long-distance running can be better treated.

## 5. Conclusion

The author proposes a method for rehabilitation monitoring of long-distance running injuries based on CT multimodal images. This method integrates multimodality technology into CT images. By medically cutting CT multimodal images and analyzing them; finally, the treatment of injuries caused by long-distance running can be achieved. Experimental results show that the method used by the author took a total of 10.9 hours, and the average time was 8 seconds, which was much shorter than the other two methods. It shows that the method of long-distance running injury rehabilitation monitoring based on CT multimodal images can effectively improve the treatment effect.

## Figures and Tables

**Figure 1:** Application of CT multimodal images in long-distance running rehabilitation monitoring.

**Figure 2:** CT values corresponding to each tissue in the human body (unit: HU).

**Figure 3:** Threshold selection based on histogram.

**Figure 4:** (a, b) show the values of *p*(*a*^*x*^|*y*_*x*_) under different intensities. *p*(*a*^*x*^|*y*_*x*_) values at different intensities.

**Table 1:** Comparison results of three methods in 110 hip joint data segmentation time.

	Zoroofi's method	Yokota's method	Our method
Total (h)	12.9	18.5	10.9
Average time (s)	9.5	13.6	8

## Data Availability

The data used to support the findings of this study are available from the corresponding author upon request.
